The article "MicroRNA-363 inhibits ovarian cancer progression by inhibiting NOB1" was retracted in 2023. Reasons: results that could not be reproduced; duplicated images.

# MicroRNA-363 inhibits ovarian cancer progression by inhibiting NOB1

**DOI:** 10.18632/oncotarget.21417

**Published:** 2017-09-30

**Authors:** Yang Lin, Tianmin Xu, Shunqing Zhou, Manhua Cui

**Affiliations:** ^1^ Department of Obstetrics and Gynecology, The Second Hospital, Jilin University, Nanguan District, Changchun 130041, China

**Keywords:** microRNAs, miR-363, ovarian cancer, NOB1

## Abstract

In this study, we investigated the role of microRNA-363(miR-363) in ovarian cancer (OC) progression. MiR-363expression was downregulated in OC patient tissues and four OC cell lines (SKOV3, A2780, OVCAR and HO-8910). Low miR-363 levels were associated with advanced stage, lymph node metastasis, and poor prognosis in OC. MiR-363 overexpression decreased growth, colony formation, migration and invasiveness of SKOV3 cells. In addition, miR-363 overexpression in SKOV3 cells also decreased xenograft tumor size and weight in nude mice. Bioinformatics and dual luciferase reporter assays revealed that miR-363 suppresses expression of NIN1/RPN12 binding protein 1 homolog (NOB1) by binding to the 3’-UTR of its transcript. NOB1 expression inversely correlated with miR-363 levels in OC tissues. Thus miR-363 appears to play a tumor suppressor role in OC by inhibiting NOB1.

## INTRODUCTION

Ovarian cancer (OC) is the most common gynecological malignancy with poor overall survival [1]. The 5-year survival rate is 35–38% despite significant improvements in therapeutic strategies for OC during the past decade [2, 3]. The underlying mechanisms that promote OC are not fully known. Therefore, elucidating novel mechanisms of OC initiation and progression are critical to developing new and improved diagnostics and therapeutics.

MicroRNAs (miRNAs) are a class of evolutionarily conserved noncoding RNAs that regulate expression of their target genes at the post-transcriptional level by binding to their 3’ untranslated region (3’UTRs) [4]. The role of miRNAs in various biological processes such as cellular proliferation, apoptosis, invasion, metastasis, migration, and stemness has been well established [5, 6]. MiRNAs perform oncogenic or tumor suppressor functions in carcinogenesis based on the function of their target proteins [7, 8]. The role of many miRNAs in the initiation, growth and metastasis of OC has already been identified [9, 10]. These miRNAs are promising prognostic biomarkers and potential therapeutic targets for OC.

MicroRNA-363 (miR-363) is a cancer-related miRNA, which plays an oncogenic or tumor suppressor role in different cancers [11–18]. However, its role in OC has remained elusive so far. Therefore, in this study, we investigated the role of miR-363 in OC progression.

The article "MicroRNA-363 inhibits ovarian cancer progression by inhibiting NOB1" was retracted in 2023. Reasons: results that could not be reproduced; duplicated images.

## RESULTS

### MiR-363 expression is decreased in OC tissues and cell lines

We determined miR-363 expression in 50 paired OC and adjacent normal tissues by qRT-PCR. OC tissues showed lower miR-363 levels than adjacent normal tissues (*p*<0.01, Figure 1A). Next, we observed lower miR-363 expression in four ovarian cancer cell lines, namely, SKOV3, A2780, OVCAR and HO-8910 than in the normal ovarian surface epithelial cell line HOSEpiC (all *p*<.05; Figure 1B). Since SKVO3 cell line showed the lowest miR-363 expression, we selected it for further study.

**Figure 1:** Low miR-363 levels correlate with OC progression **(A)** qRT-PCR analysis of miR-363 in 50 paired OC and adjacent normal tissues. **(B)** qRT-PCR analysis of miR-363 in four human ovarian cancer cell lines, SKOV3, A2780, OVCAR and HO-8910 and a human ovarian surface epithelial cell line, HOSEpiC. **(C)** Kaplan-Meier survival curve analysis demonstrates decreased 5year survival in patients expressing low levels of miR-363. Note: ^*^ denotes *p*<0.05; ^**^ denotes *p*<0.01.

### Low miR-363 levels correlate with poor prognosis of OC patients

Next, we determined the prognostic significance of miR-363 in OC. We divided patients into miR-363 low and miR-363 high groups using the median value of 0.36 as a cut off value. As shown in Table 1, low miR-363 expression was associated with advanced FIGO stage and lymph node metastasis (both *p*<0.01), but was not associated with patient age, histological grading, or tumor size (all *p*>0.05). Kaplan Meier analyses indicated that patients with low miR-363 expression were associated with reduced 5-year overall survival (*p*<0.001, Figure 1C). Thus, miR-363 demonstrates potential as a prognostic biomarker for OC patients.

**Table 1:** Association between miR-363 expression and clinicopathological features of human ovarian cancer

Variables	No. of cases	miR-363 expression		*p* value
		Low (n %)	High (n %)	
**Age(years)**				*p*>0.05
<60	22	13(59.1)	9(40.9)	
≥60	28	16(57.1)	12(42.9)	
**Tumor size**				*p*>0.05
<5 cm	35	21(60.0)	14(40.0)	
≥5 cm	15	8(53.3)	7(46.7)	
**FIGO stage**				*p*<0.05
I-II	33	14(42.4)	19(57.6)	
III-IV	17	15(88.2)	2(11.8)	
**Histological grading**				*p*>0.05
1-2	31	17(54.8)	13(45.2)	
3	19	12(63.2)	8(46.7)	
**Lymph node metastasis**				*p*<0.01
No	39	19(48.7)	20(51.2)	
Yes	11	10(90.9)	1(9.1)	

### MiR-363 overexpression inhibits OC cell proliferation and xenograft tumor growth

To investigate the biological function of miR-363 in OC, we generated control or miR-363 overexpressing SKOV3 cells with lentiviruses carrying hsa-miR-363 or has-miR-NC (Figure 2A). CCK8 assay demonstrated that miR-363 overexpression inhibited SKOV3 cell proliferation (*p*<0.05; Figure 2B). Moreover, miR-363 decreased the number of colonies (*p*<0.05; Figure 2C).

The article "MicroRNA-363 inhibits ovarian cancer progression by inhibiting NOB1" was retracted in 2023. Reasons: results that could not be reproduced; duplicated images.

**Figure 2:** MiR-363 inhibits OC cell proliferation and reduces xenograft tumor growth in nude mice **(A)** qRT-PCR analysis of miR-363 expression inmiR-363 and miR-NC transfected SKOV3 cells. **(B)** CCK8 assay showing cell proliferation rates of miR-363 and miR-NC transfected SKOV3 cells. **(C)** Estimation of colonies in SKOV3 cells stable expressing miR-363 and miR-NC. **(D)** Xenograft tumor volumes in nude mice injected with SKOV3 cells stable expressing miR-363 and miR-NC. Tumor volumes were measured every 5 days until day 30 when mice were sacrificed. **(E)** Representative images of xenograft tumors derived from SKOV3 cells stable expressing miR-363 and miR-NC. Note: ^*^ denotes *p*<0.05;^**^ denotes *p*<0.01.

To determine the significance of these findings *in vivo*, SKOV3 cells stable expressing miR-363 or miR-NC were subcutaneously injected into the flank region of nude mice. We observed decreased tumor growth in the miR-363 group than in the miR-NC group (*p*<0.05, Figure 2D). When the xenografted tumors were harvested on day 30, we observed decreased tumor size in miR-363 group than the miR-NC group (*p*<0.05, Figure 2E). These data demonstrate that miR-363 inhibits OC growth and progression.

### MiR-363 suppresses OC cell migration and invasion

Next, we investigated the role of miR-363 in OS metastasis. MiR-363 overexpressing SKOV3 cells showed decreased migration and invasiveness than control cells (both *p*<0.01; Figure 3A-3B).

**Figure 3:** MiR-363 inhibitsovarian cancer cell migration and invasion **(A)** Wound healing assay showing migration of control and miR-363 overexpressing SKOV3 cells. **(B)** Transwell assay showing invasiveness of control and miR-363 overexpressing SKOV3 cells. Note: ^*^ denotes *p*<0.05;^**^ denotes *p*<0.01.

### NOB1 is a target of miR-363 in OC cells

We explored Targetscan and miRanda websites and identified *NOB1* as the potential miR-363 target gene with a probable binding site at bases 217 to 223 (Figure 4A). We performed dual luciferase reporter assays in control or miR-363 overexpressing SKOV3 cells transfected with wild type or mutant NOB1-3’UTR. As shown in Figure 4B, miR-363 overexpressing SKOV3 cells transfected with the WT-NOB1-3’UTR construct showed decreased luciferase activity than miR-363 overexpressing SKOV3 cells transfected with the mutant NOB1-3’UTR construct. Moreover, miR-363 ovexpression decreased NOB1 mRNA and protein expression (Figure 4C-4D).

**Figure 4:** NOB1 is the miR-363target in SKOV3ovarian cancer cells **(A)** Sequence alignment of putative wild-type (WT) and mutant (MT) miR-363-binding sites in the 3’-UTR of *NOB1*. **(B)** Dual luciferase reporter assay showing decreased luciferase activity in SKOV3 cells overexpressing miR-363 in combination with wild type NOB1-3’UTR than in SKOV3 cells overexpressing miR-363 in combination with mutant NOB1-3’UTR. **(C)** qRT-PCR analysis of *NOB1* mRNA levels in control and miR-363 overexpressing SKOV3 cells. **(D)** Western blot analysis of NOB1 protein levels in control and miR-363 overexpressing SKOV3 cells. Note: ^*^ denotes *p*<0.05;^**^ denotes *p*<0.01.

The article "MicroRNA-363 inhibits ovarian cancer progression by inhibiting NOB1" was retracted in 2023. Reasons: results that could not be reproduced; duplicated images.

### NOB1 mediates the functional effects of miR-363 on OS cells

We observed that co-transfection of SKOV3 cells with miR-363 mimics and NOB1 overexpressing plasmid restored NOB1 levels in SKOV3 cells (Figure 5A-5B). Increased NOB1 levels restored SKOV3 cell proliferation, colony formation, migration and invasion (Figure 5C-5F). These data demonstrated that miR-363 inhibits OC cell growth and metastasis by decreasing NOB1 expression.

**Figure 5:** NOB1 expression regulates OS progression **(A)** qRT-PCR analysis of NOB1 mRNA levels in SKOV3 cells co-transfected with NOB1 plasmid without 3’UTR in combination with either miR-363 mimic or miR-NC. GAPDH was used as an internal control. **(B)** Western blot analysis of NOB1 protein levels in SKOV3 cells co-transfected with NOB1 plasmid without 3’UTR in combination with either miR-363 mimic or miR-NC. **(C)** CCK8 assay showing cell proliferation in SKOV3 cells co-transfected with NOB1 plasmid without 3’UTR in combination with either miR-363 mimic or miR-NC. **(D)** Estimation of number of colonies in SKOV3 cells stable expressing miR-363 or miR-NC transfected with NOB1 plasmid without 3’UTR. **(E)** Wound healing assay estimating migration of SKOV3 cells co-transfected with NOB1 plasmid without 3’UTR in combination with either miR-363 mimic or miR-NC. **(F)** Transwell assay estimating invasiveness of SKOV3 cells co-transfected with NOB1 plasmid without 3’UTR in combination with either miR-363 mimic or miR-NC. Note:^*^ denotes *p*<0.05;^**^ denotes *p*<0.01.

### NOB1 inversely correlates with miR-363 in OC tissues

Next, we investigated the relative expression of NOB1 mRNA and miR-363 in 50 pairs of OC and corresponding adjacent normal tissues by qRT-PCR. *NOB1* mRNA levels were higher in the OC tissues than the adjacent normal tissues (*p*<0.05; Figure 6A). Immunohistochemical analysis demonstrated higher NOB1 protein expression in OC tissues than the adjacent normal tissues (Figure 6B). Moreover, Spearman's rank test showed that *NOB1* transcript levels inversely correlated with miR-363 expression (r=-0.659, *p*<0.001, Figure 6C).

**Figure 6:** NOB1 expression inversely correlates with miR-363 levels in patient OC tissues **(A)** qRT-PCR analysis of *NOB1* mRNA expression in 50 paired OC and adjacent normal tissues. GAPDH was used as an internal control. **(B)** Immunohistochemical analysis of NOB1 protein expression in OC tissue samples. **(C)** Spearman's correlation analysis of the association between the NOB1 and miR-363 expression in human ovarian cancer (n=50). Note: ^*^ denotes *p*<0.05;^**^ denotes *p*<0.01.

The article "MicroRNA-363 inhibits ovarian cancer progression by inhibiting NOB1" was retracted in 2023. Reasons: results that could not be reproduced; duplicated images.

## DISCUSSION

MicroRNAs (miRNAs) play crucial roles in ovarian cancer progression [19, 20]. In this study, we investigated the role of miR-363 in OC progression. We found significant downregulation of miR-363 in OC tissues and cell lines than normal ovarian tissues and cell line, respectively. Moreover, decreased miR-363 levels correlated with poor prognosis of OC. MiR-363 overexpression inhibited cellular proliferation, colony formation, migration and invasion. The miR-363 overexpressing OC cells decreased xenograft tumor growth resulting in smaller tumors in nude mice. MiR-363 inhibited OC cell proliferation and progression by inhibiting NOB1 expression.

The role of miR-363 has focused on cancer diagnosis and treatment. It acts as a tumor suppressor in thyroid [21], head and neck [12], colorectal [13], head and neck [17], breast [16], and renal [14] cancers. In contrast, miR-363 plays an oncogenic role in prostate [18], and gastric [12] cancers. This demonstrates conflicting roles of miR-363 in different cancers. However, the status and role of miR-363 in OC progression is not known. Our study demonstrates tumor suppressor function for miR-363 in OC. Bioinformatics analysis identified *NOB1* as a potential target gene of miR-363 based on its role and expression in ovarian cancer. *NOB1* is a 50 kDa protein subunit of the 26S proteasome complex consisting of PIN and zinc ribbon domains [22]. It is necessary for the function of the 26S proteosomal function [23]. NOB1 expression is upregulated in cervical [24], gastric [25], laryngeal [26], lung [27] prostate [28], and thyroid [29]. NOB1 expression is upregulated in ovarian cancer tissues and its knockdown decreased cell proliferation, colony formation and induced G1-S cell cycle arrest [30].Moreover, it increased TRAIL sensitivity in ovarian cancer cells [31]. MiR-215 inhibited *in vitro* ovarian cancer cell proliferation, colony formation, migration and invasion, as well as *in vivo* tumor growth by targeting *NOB1* [32]. These results suggested oncogenic role for NOB1 in ovarian cancer. In this study, we identified NOB1 as a target of miR-363. Overexpression of NOB1 partially abrogated the suppression effect on proliferation, colony formation, migration and invasion of OC cells induced by miR-363. Moreover, OC patient samples demonstrated an inverse relationship between NOB1 and miR-363 expression. These data indicated that miR-363 performed tumor suppressor function in ovarian cancer cells by targeting NOB1.

The article "MicroRNA-363 inhibits ovarian cancer progression by inhibiting NOB1" was retracted in 2023. Reasons: results that could not be reproduced; duplicated images.

The main limitation of our study is that we analyzed fewer OC patient samples and cell types. Therefore, more elaborate studies are necessary for further explore the potential therapeutic and prognostic role of miR-363 in OC progression. In conclusion, our results demonstrate that miR-363 functions as a tumor suppressor in OC by targeting NOB1 in OC and represents a potential therapeutic target for OC treatment.

## MATERIALS AND METHODS

### Clinical samples

Fifty pairs of cancer and adjacent normal tissues (>3 cm from cancer tissue) were obtained from 50 OC patients (Mean 61.7 years) that underwent surgical resection at the Department of Obstetrics and Gynecology, The Second Affiliated Hospital of Jilin University, Changchun, China. The tissue samples were snap frozen and stored in liquid nitrogen for further investigation. We excluded patients that received immunotherapy, chemotherapy or radiotherapy before surgical treatment. The disease stages were classified according to the International Federation of Obstetrics and Gynecology (FIGO) criteria. The demographic features and clinicopathological characteristics of all patients are listed in Table 1. Informed consent was signed by each patient before surgery. This study was approved by the Research Ethics Committee of our institute.

### Cell lines and cell culture

The four human ovarian cancer cell lines, SKOV3, A2780, OVCAR and HO-8910, and the human ovarian surface epithelial cell line, HOSEpiC were obtained from Chinese Academy of Sciences, Shanghai, China. All cell lines were grown in RPMI-1640 medium (Gibco-BRL, Gaithersburg, MD, USA) supplemented with 10% fetal bovine serum ( FBS; HyClone, Logan, Utah, USA) and 1% penicillin/streptomycin at 37 °C and 5% CO_2_.

### Transfection studies

Lentiviral vector pGreenPuro (System Biosciences, USA) with hsa-miR-363(miR-363) or hsa-miR-negative control (miR-NC) was packaged in 293T cells using the lentiviral packaging kit (GeneCopoeia, Shanghai, China) according to manufacturer's manual. Stable cell lines were established by infecting SKOV3 cells with lentiviruses encoding miR-363 or miR-NC followed by 2 mg/ml puromycin selection. The stable cell lines were cultured in RPMI-1640 medium containing 10% FBS and puromycin (0.5 mg/ml) for colony formation assay and *in vivo* experiments. The miR-363 mimic and the corresponding negative control, miR-NC was brought from GenePharma (Shanghai, China). The NOB1 overexpression vector (pCDNA3.1-NOB1) without 3’ UTR was constructed as previously described [32]. miR-363 mimic, miR-NC, or pCDNA3.1-NOB1 plasmid were transfected into cells using Lipofectamine™ 3000 reagent (Invitrogen, Carlsbad, CA, USA) according to manufacturer's protocol.

The article "MicroRNA-363 inhibits ovarian cancer progression by inhibiting NOB1" was retracted in 2023. Reasons: results that could not be reproduced; duplicated images.

### Quantitative real-time PCR

Total RNA was prepared from the tissue samples and cultured cells with TRIzol reagent (Invitrogen) according to manufacturer's manual. The relative expression of miRNA-363 was detected using a SYBR PrimeScript miRNA RT PCR kit (Takara, Dalian, China) in accordance with the manufacturer's instructions. For detection of *NOB1* mRNA expression, first-strand cDNA synthesis was performed with MMLV reverse transcriptase (Promega, USA) according to the manufacturer′s instructions. Real time PCR was performed using SYBR Premix Ex Taq (TaKaRa, Dalian, China) in a ABI 7900 Fast system (Applied Biosystems, CA, USA). miR-363 and U6 primers were purchased from Applied Biosystems. The primers for NOB1 and GAPDH were as described in previous studies [29]. The relative expression of miR-363 and NOB1 were normalized to U6 and GAPDH levels, respectively using the 2^-ΔΔCT^method.

### Cell proliferation

We determined cell proliferation using the Cell Counting Kit-8(CCK8) assays. Briefly, 2 × 10^3^ transfected cells were seeded into 96-well plates and cultured at 5% CO_2_ and 37°C for 24 -72 h. At each time point, 10μl of CCK-8 solution(Dojindo Laboratories, Kumamoto, Japan) was added and the cells were further incubated for 1 h. The absorbance was read at 450 nm was in a microplate reader (Bio-Tek Company, Winooski, VT, USA).

### Colony formation assay

The SKOV3-miR-363 and SKOV3-miR-NC cells (500 cells/well) were cultured in six-well plates for 14 days. Then, the colonies were fixed in 20% methanol and stained with 0.5 % crystal violet for 15 min. The number of colonies were determined after imaging in a light microscope (Olympus, Tokyo, Japan).

### Cell migration and invasion assays

To determine migratory ability of OC cells, wound healing assays were performed by growing transfected cells (1×10^5^/well) to confluence in 6-well plates. Subsequently, the cells were scratched with a sterile plastic micropipette tip to generate an homogenous wound in the monolayer. The cells were washed with PBS and cultured under standard conditions for 24 h. Then, the cells were imaged at 0 and 24 h after the wounding with an inverted Nikon Eclipse TS100 phase-contrast microscope (Tokyo, Japan). Wound closure was measured with the Nikon NIS-Element Basic Research v3.2 software (Tokyo, Japan).

Cell invasiveness was determined using Transwell assay. Briefly, 2×10^5^ cells in serum-free media were seeded into the upper chamber that is coated with matrigel. In the lower chamber, RPMI 1640 medium with 20% FBS was added as a chemoattractant. After 24 h, the non-invading cells were gently removed with a cotton swab, whereas cells that invaded the lower surface of the filter were fixed with 70% ethanol for 30 min and stained with 0.1% crystal violet for 10 min. The cells were photographed with an inverted light microscope (Zeiss, Germany) at 200x magnification and the cell numbers were counted in five random fields of view.

The article "MicroRNA-363 inhibits ovarian cancer progression by inhibiting NOB1" was retracted in 2023. Reasons: results that could not be reproduced; duplicated images.

### Dual-luciferase reporter assay

The 3′-untranslated region (3’-UTR) of NOB1 with the potential binding sites of miR-363 (position 217-223) was PCR amplified and subcloned into psiCHECK2 vector (Promega, Wisconsin, WI, USA). It is referred to as WT-NOB1-3’UTR. The mutant 3’-UTR of NOB1 was constructed with QuikChange XL Site-Directed Mutagenesis Kit (Agilent Technologies; Santa Clara, CA) and subcloned into psiCHECK2 vector. It is referred to as MT-NOB1-3’UTR. For the luciferase reporter assay, SKOV3 cells were grown to 70-80% confluence and transfected with miR-363 mimic or miR-NC in combination with WT-NOB1-3’-UTR or MT-NOB1-3’-UTR. The firefly and renilla luciferase activities were determined using the Dual-Luciferase Reporter Assay System (Promega). The ratio of firefly to renilla luciferase activities were used to determine if miR-363 regulated NOB1 expression by binding to its 3’UTR.

### Western blotting

Protein extraction and western blotting were performed as previously described [31]. Briefly, cultured cells or tissues were harvested and lysed with RIPA buffer (Beyotime, Jiangsu, China), following by quantification with BCA protein assay kit (Pierce, Bonn, Germany). Protein samples were fractionated by 10% SDS- PAGE, the proteins were blotted onto nitrocellulose membrane (Amersham BioSciences, Buckinghamshire, UK). The membranes were immunoblotted with antibodies against NOB1 (Santa Cruz Biotechnology, Santa Cruz, CA, USA) and GAPDH (Santa Cruz Biotechnology), followed by HRP-linked secondary antibodies (Santa Cruz Biotechnology). The protein band were detected by SuperSignal West Pico Chemiluminescent Substrate kit (Pierce, Rockford, IL, USA). GAPDH was used as a control.

### Immunohistochemistry (IHC)

Formalin-fixed and paraffin-embedded tumor tissues were cut into 4 μm sections. Then, paraffin sections were deparaffined in xylene and dehydrated in graded ethanol. Heat induced antigen retrieval were performed using Citrate buffer(Invitrogen). Non-specific antibody binding were blocked by with 5% skimmed milk. Then, sections were incubated with the primary anti-NOB1 antibody (1:400, Santa Cruz Biotechnology) overnight at 4°C. Thefollowing day, the slides were incubated with horseradish peroxidase conjugatedsecondary antibody (ZSGB BIO, Beijing China) for 90 min at room temperature, and aperoxidase-labeled polymer for 10 min at room temperature. The slides were developed with freshly prepared DAB solution for 5 min followed by hematoxylin counterstain. Then, after dehydration and mounting, they were photographed under a light microscope. The NOB1 positive cells were calculated as described previously [29].

The article "MicroRNA-363 inhibits ovarian cancer progression by inhibiting NOB1" was retracted in 2023. Reasons: results that could not be reproduced; duplicated images.

### *In vivo* xenograft study

Animal study was approved by the Committee on the Use of Live Animals in Teaching and Research of the Animal Research Committee Jilin University, Changchun, China. Tumor xenograft model was established in 6 week old female BALB/c nu/nu mice (Experimental Animal Center of the Jilin University, Changchun, China) by subcutaneously injecting 2×10^6^ SKOV3 cells expressing miR-363 or miR-NC into the flank region (n=10 per group). Tumor growth was monitored every 5 days with a fine digital caliper by measuring tumor length(L) and width(W). Tumor volume was calculated as (L × W^2^)/2. After 30 days, mice were killed, and the tumors were harvested and weighed.

### Statistical analysis

Statistical Package of the Social Sciences 17.0 for Windows (SPSS, Chicago, IL, USA) was used for statistical analyses. The data shown are presented as the mean ±SD (standard deviation) at least from three independent experiments. Differences between experimental groups were analyzed by Student's *t* test when only two groups were compared and Tukey's one-way ANOVA when more than two groups were compared. The relationship between miR-363 and NOB1 expression was assessed by Spearman's correlation analysis. A *p* value less than 0.05(*p*<0.05) was considered statistically significant.
